This article has been retracted.

# Protective Role of Amiodarone on Reperfusion Arrhythmia in Patients of Acute Myocardial Infarction with Percutaneous Coronary Intervention Treatment

**DOI:** 10.1155/2022/2597173

**Published:** 2022-08-26

**Authors:** Jianying Wang, Jinchang Leng, Xiaowei Sun, Kun Peng, Xaojuan Ma, Shiqin Huang, Fang Wang

**Affiliations:** ^1^Department of Infomation, Medical Supplies Center of PLA General Hospital, Beijing 100039, China; ^2^Department of Pharmacy, Medical Supplies Center of PLA General of PLA General Hospital, Beijing 100039, China

## Abstract

With the development and popularity of percutaneous coronary intervention (PCI), ischemia-reperfusion injury (IRI) has attracted more and more clinical attention. Reperfusion arrhythmia (RA), one of the common manifestations during and after PCI, can affect the postoperative cardiac function of patients with acute myocardial infarction (AMI). Therefore, effective intervention on RA has important clinical significance. This study observed the effect of amiodarone on reperfusion arrhythmia (RA) after percutaneous coronary intervention (PCI) in patients with acute myocardial infarction (AMI) and explored its possible mechanism. The results showed that amiodarone had good clinical efficacy in the prevention of RA in patients with AMI after PCI, and it could reduce the levels of serum IL-6, hs-CRP, CK-MB, and cTnI in patients and reduce the damage caused by reperfusion, thereby reducing the occurrence of RA.

## 1. Introduction

Percutaneous coronary intervention (PCI) is currently the most important method for the treatment of acute myocardial infarction (AMI). However, after vascular recanalization, it will cause ischemia-reperfusion injury (IRI) to the myocardium, resulting in arrhythmia, heart failure, cardiogenic shock, and other symptoms, which seriously affect the prognosis of patients with AMI [1]. Reperfusion arrhythmia (RA), as one of the common manifestations during and after PCI, has an impact on the recovery of postoperative cardiac function, and prevention of this disease will help to improve the prognosis of patients and restore cardiac function [2]. Amiodarone multichannel blockers have the pharmacological effects of all antiarrhythmic drugs in class I to IV, as well as mild noncompetitive *α* and *β*-adrenergic receptor blockade and mild antiarrhythmic drugs in class I and class IV [3]. In clinical practice, amiodarone not only has a certain effect on the ventricular premature beat, ventricular tachycardia, and ventricular fibrillation after myocardial infarction and heart failure but also has a certain effect on reducing mortality [4]. Therefore, this study aimed to observe the effect of preoperative amiodarone on postoperative RA in patients with AMI undergoing emergency PCI and to explore its mechanism.

## 2. Materials and Methods

### 2.1. Research Objects

According to the following inclusion and exclusion criteria, patients with AMI who received emergency PCI in our hospital from August 2017 to February 2018 were selected as the research subjects. After review and approval by the hospital ethics committee, a total of 264 patients with AMI were included in this study, and the patients were randomly divided into the control group (conventional PCI group) with 132 cases and the study group (amiodarone intervention group) with 132 cases according to the random number table method. The clinical data of the patients and the number of diseased coronary arteries and infarct sites were recorded.

### 2.2. Inclusion Criteria

Inclusion criteria are as follows: (1) meet the diagnostic criteria of the Chinese Medical Association for AMI [5]; (2) perform PCI within 24 hours after onset; (3) Killip grade 1–2; (4) sinus rhythm, and before treatment not taking antiarrhythmic drugs; and (5) the patient's family signed informed consent.

### 2.3. Exclusion Criteria

Exclusion criteria are as follows: (1) with mechanical complications such as ventricular septal perforation and valve prolapse; (2) with severe systemic diseases; (3) with peripheral vascular disease and aortic aneurysm; (4) with coagulation disorders etc.; (5) there was bradyarrhythmia before treatment; (6) a pacemaker had been installed; and (7) proximal right coronary artery occlusion.

### 2.4. Treatment Methods

All patients received emergency PCI, while the control group received conventional treatment, including aspirin, clopidogrel or ticagrelor, beta-blockers, and statins. On the basis of the conventional PCI group, the amiodarone intervention group was given amiodarone hydrochloride injection before the operation, and the injection was continuously pumped at the speed of 1 mg/min until 4 hours after the operation. If there was tachycardia and the blood pressure dropped during the treatment, the infusion was stopped.

Interventional treatment methods: preoperative aspirin 300 mg plus clopidogrel 600 mg or ticagrelor 180 mg, coronary angiography via the femoral artery or radial artery, and unfractionated heparin if the infarct-related vascular (IRA) lesions are clearly shown. Stents were placed directly after 100 U/kg anticoagulation, and stents were placed after balloon dilation for subtotal occlusion or total occlusion of IRA. TIMI blood flow grade III with lumen stenosis <30% indicates successful stent placement. After the operation, the patients continued to take dual antibacterial drugs, were routinely given statins and other drugs, and were given ACEI or *β*-blockers according to their condition.

### 2.5. Observation Indicators

#### 2.5.1. Occurrence of Reperfusion Arrhythmia

The patients received continuous ECG monitoring during and after the operation, and the observation time for RA was within 4 hours after the opening of IRA. More than one min, tachyarrhythmias such as ventricular premature beats, ventricular tachycardia, atrial fibrillation, and ventricular fibrillation occur [6].

#### 2.5.2. Laboratory Examination

5 ml of fasting venous blood was drawn from all patients at the time of admission and 24 hours after the operation. The levels of high-sensitivity C-reactive protein (hs-CRP) and interleukin -6 (IL-6) were detected by nephelometry and enzyme-linked immunosorbent assay (ELISA). The myocardial troponin I(cTnI) level was detected by the chemiluminescence method. The creatine kinase isoenzyme (CK-MB) level was detected by the rate method.

### 2.6. Statistical Methods

Statistical analysis was performed using SPSS 22.0 software. Measurement data were expressed as mean ± standard deviation ($\bar{x}\pm S$). If it conformed to normal distribution and homogeneity of variance, the *t*-test was used for comparison between the two groups; if it did not conform to normal distribution, the rank sum test was used. Enumeration data were expressed as absolute numbers or percentages (%), and the *χ*^2^ test or rank sum test was used. Differences were considered significant at *P* < 0.05.

## 3. Results

### 3.1. Comparison of General Data of the Two Groups of Patients

In the routine PCI group, there were 84 males (63.6%) and 48 females (36.4%), with an average age of 59.3 ± 8.0 years and a body mass index (BMI) of 24.2 ± 3.5 kg/m^2^; the amiodarone intervention group included 87 males (65.9%) and 45 females (34.1%), with an average age of 57.6 ± 6.6 years and a body mass index of 24.8 ± 2.4 kg/m^2^. There were no significant differences in age, gender, BMI, history, infarct location, and number of stenotic or occluded coronary branches between the two groups of AMI patients (*P* > 0.05), as shown in Table 1.

### 3.2. The  Occurrence of Reperfusion Arrhythmia

A total of 137 cases (51.9%) of RA occurred after PCI, including 89 cases (67.4%, 89/132 cases) in the conventional PCI group and 48 cases (36.4%, 48/132 cases) in the amiodarone intervention group. Ventricular arrhythmias are most common, ventricular tachycardia and ventricular premature beats are more common, and bradyarrhythmias and ventricular fibrillation are rare. Compared with the conventional PCI group, the incidence of RA in the amiodarone intervention group was lower, and the difference was significant (*P* < 0.01). Among them, the incidence of ventricular fibrillation and defibrillation in the intervention group was lower than that in the conventional group. In addition, the incidence of premature ventricular contractions and ventricular tachycardia in the intervention group was also lower than that in the conventional PCI group, and the differences were statistically significant (*P* < 0.05). Bradyarrhythmia were rare in both groups, with 18 (13.6%) and 12 (9.1%), respectively, as shown in Table 2.

### 3.3. Laboratory  Tests

After PCI, the levels of serum IL-6 and hs-CRP in the two groups were increased compared with those before treatment, while the levels of cTnI and CK-MB were decreased compared with those before treatment, and the difference was statistically significant (*P* < 0.05). Compared with the control group, the levels of IL-6, hs-CRP, cTnI, and CK-MB in the amiodarone intervention group were significantly lower after treatment, and the difference was statistically significant (*P* < 0.05), as shown in Table 3.

## 4. Discussion

As a common treatment for AMI, PCI can open narrowed or occluded blood vessels, increase myocardial blood supply, and significantly improve myocardial diastolic and systolic function [7]. However, while blood reperfusion increases blood supply, it may also aggravate myocardial damage and cause IRI, which manifests as severe or even fatal arrhythmia, heart failure, or cardiogenic shock [8]. With the development and popularization of PCI, IRI has received more and more clinical attention, but its mechanism has not yet been fully clarified. Studies have shown that calcium ion overload, the production of a large number of oxygen free radicals, and the secretion of endothelial factors by vascular endothelial cells may be related to this pathophysiological process [9]. In addition, the activation of neutrophils, the increase of myocardial automaticity, and the Vf threshold of ischemic myocardium, the decline of myocardial electrolytes, myocardial electrolyte disturbance, etc. may be involved in the occurrence of IRI [10]. RA is one of the common manifestations of IRI. The occurrence of RA will not only aggravate the damage to the ischemic myocardium but also have a serious impact on hemodynamics. If it is not terminated in time, it may lead to further deterioration of cardiac function and further increase the mortality rate. Therefore, early treatment and prevention of ventricular arrhythmia after myocardial infarction has become an important measure to reduce its mortality [11]. Therefore, effective intervention for RA has important clinical significance.

Amiodarone is a class III antiarrhythmic drug that can delay ischemic myocardial conduction and reduce the action potential of ischemic and nonischemic myocardium, thereby reducing reentrant excitation and triggered activity and helping to inhibit the occurrence of arrhythmia [12]. Clinical studies have shown that in acute myocardial ischemia or myocardial infarction, amiodarone can increase the activity of ion channels without aggravating the deterioration of cardiac function and has no effect on myocardial ischemia [13, 14]. All kinds of arrhythmia combined in the blood have a better effect. In this study, the incidence of RA in the conventional PCI group and the amiodarone intervention group was 67.4% and 36.4%, respectively. The incidence of RA in the AMI patients with amiodarone intervention was significantly lower, and the proportion of various ventricular arrhythmias, especially the occurrence of ventricular fibrillation, was significantly lower than that of the conventional group. This suggests that amiodarone has a better preventive effect on the occurrence of RA, especially ventricular arrhythmia, thereby reducing the risk of ventricular tachycardia.

In IRI, amiodarone not only acts as an antiarrhythmic but also protects cardiomyocytes [15]. After the occurrence of AMI, the permeability of the myocardial cell membrane increases, causing the intracellular CK-MB and cTnI to leak out, resulting in an increase in the concentration of CK-MB and cTnI in the blood of patients, so the levels of the two are more sensitive indicators to reflect the degree of myocardial injury [16]. Animal experiments have shown that amiodarone can reduce serum CK-MB and cTnI levels in rats with myocardial ischemia-reperfusion, suggesting that it can alleviate acute myocardial ischemia-reperfusion injury in rats [17]. In this study, the serum cTnI and CK-MB levels in the amiodarone intervention group after PCI were significantly lower than those in the routine PCI group, suggesting that in patients with AMI undergoing emergency PCI, the use of amiodarone intervention can reduce myocardial injury.

Activation of neutrophils is an important pathway for IRI. IL-6 is a cytokine that mediates inflammatory responses, and inhibiting the release of inflammatory factors can reduce the accumulation of neutrophils in microvessels, thereby reducing myocardial damage [18]. In addition, according to research, hs-CRP content was significantly negatively correlated with the prognosis of PCI patients [19]. In this study, the levels of serum IL-6 and hs-CRP in patients after PCI were higher than those before treatment, indicating that reperfusion activated neutrophils and caused a large number of inflammatory factors to be released. The levels of serum IL-6 and hs-CRP in AMI patients treated with amiodarone after PCI were significantly lower than those in the conventional PCI group, indicating that amiodarone can improve the level of inflammatory factors, thereby effectively reducing IRI. In addition to the above mechanisms, amiodarone also can inhibit Na^+^/Ca^2+^ exchange protein, thereby reducing calcium overload during blood reperfusion.

In conclusion, amiodarone can protect ischemic myocardium in various ways. Preoperative amiodarone intervention in patients with AMI can reduce the levels of serum IL-6, hs-CRP, CK-MB, and cTnI after PCI, reduce the damage caused by reperfusion, thereby reducing the occurrence of RA and providing a basis for preventing the occurrence of RA after PCI [20].

## Figures and Tables

**Table 1:** Comparison of the general conditions of the two groups of patients ($\bar{x}\pm S$, *n* (%)).

General conditions	Regular PCI group (*n* = 132)	Amiodarone intervention group (*n* = 132)	*χ * ^2^/*t* value	*P* value
Age (year)	59.3 ± 8.0	57.6 ± 6.6	1.883	0.061
Gender (male)	84 (63.6)	87 (65.9)	0.149	0.699
Body mass index (kg/m^2^)	24.2 ± 3.5	24.8 ± 2.4	−1.624	0.106
Diabetes	61 (46.2)	64 (48.5)	0.137	0.712
Hypertension	98 (74.2)	91 (68.9)	0.913	0.339
Hyperlipidemia	73 (55.3)	70 (53.0)	0.137	0.711
History of smoking	88 (66.7)	91 (68.9)	0.156	0.693
Infarct site				
Extensive, anterolateral sidewall	114 (86.4)	119 (90.2)	0.914	0.339
Inferior wall, posterior wall, right ventricle	18 (13.6)	13 (9.8)		
The number of coronary arteries with lesions				
1 artery	71 (53.8)	75 (56.8)	5.158	0.161
2 arteries	41 (31.1)	38 (28.8)		
3 arteries	20 (15.2)	19 (14.4)		

**Table 2:** Comparison of the incidence of reperfusion arrhythmia in the two groups of patients (*n*, %).

	Regular PCI group (*n* = 132)	Amiodarone intervention group (*n* = 132)	*χ * ^2^ value	*P* value
Incidence of arrhythmia	89 (67.4)	48 (36.4)	25.506	<0.001
Premature ventricular contractions	29 (22.0)	16 (12.1)	4.527	0.033
Ventricular tachycardia	22 (16.7)	11 (8.3)	4.190	0.041
Ventricular fibrillation	10 (7.6)	2 (1.5)	5.587	0.018
Sinus bradycardia	11 (8.3)	7 (5.3)	0.954	0.329
High-grade atrioventricular block	7 (5.3)	5 (3.8)	0.349	0.555
Various cardiac arrhythmias	10 (7.6)	7 (5.3)	0.566	0.452

**Table 3:** Comparison of serum IL-6, hs-CRP, cTnI, and CK-MB levels in the two groups of patients before and after treatment ($\bar{x}\pm S$).

Group	Time	IL-6 (pg/ml)	Hs-CRP (mg/L)	cTnI (ng/mL)	CK-MB (U/L)
Regular PCI group (*n* = 132)	Before treatment	4.09 ± 0.36	7.02 ± 1.03	13.11 ± 2.02	243.15 ± 21.46
	After treatment	5.05 ± 0.31^△^	8.12 ± 1.20^△^	8.43 ± 1.85^△^	186.67 ± 25.32^△^

Amiodarone intervention group (*n* = 132)	Before treatment	4.01 ± 0.42	7.23 ± 1.05	12.98 ± 2.10	245.92 ± 23.17
	After treatment	4.76 ± 0.29^*∗*^^△^	7.64 ± 1.12^*∗*^^△^	6.31 ± 1.79^*∗*^^△^	112.33 ± 27.83^*∗*^^△^

*Note.* Compared with the conventional PCI group after treatment, ^*∗*^*P* < 0.05; compared with the same group before treatment, ^Δ^*P* < 0.05.

## Data Availability

The raw data supporting the conclusion of this article will be available by the corresponding author without undue reservation.
